The article "Application of Pet-CT Fusion Deep Learning Imaging in Precise Radiotherapy of Thyroid Cancer" was published in 2021. Journal: J Healthc Eng.

# Application of Pet-CT Fusion Deep Learning Imaging in Precise Radiotherapy of Thyroid Cancer

**DOI:** 10.1155/2021/2456429

**Published:** 2021-08-05

**Authors:** Qiuyu Lin, Qianle Qi, Sen Hou, Zhen Chen, Nan Jiang, Lan Zhang, Chenghe Lin

**Affiliations:** ^1^Nuclear Medicine Department, The First Hospital of Jilin University, Changchun 130000, Jilin, China; ^2^Chengdu Xinke Pharmaceutical Co. Ltd., Chengdu 610000, Sichuan, China; ^3^Biological Sciences, Cornell University, Ithaca 14850, NY, USA

## Abstract

This article explores the value of wall F-FDG PET/Cr imaging in the diagnosis of thyroid cancer, studies its ability to distinguish benign and malignant thyroid lesions, and seeks ways to improve the accuracy of diagnosis. The normal control group selected 40 patients who came to our center for physical examination. In the normal control group, the average value of the standard uptake value of both sides of the thyroid was used as the SUV of the thyroid gland and the highest SUV value of the patient's lesion (SUV max) represented the SUV of the lesion. After injection of imaging agent 18F-FD1G, routine imaging was performed at 1h, time-lapse imaging was performed at 2.5 h, and the changes with conventional imaging were compared to infer the benign and malignant lesions. We used SPSS software to carry out statistical analysis, respectively, carrying out analysis of variance, paired *t*-test, independent sample *t*-test, and linear correlation analysis. In the thyroid cancer group, 87.5% of the delayed imaging SUV was higher than the conventional imaging SUV, while 83.33% of the benign disease group had a lower SUV than the conventional imaging SUV. 18F-FDG PET/CT imaging has higher sensitivity and specificity for the diagnosis of recurrence or metastasis in patients with Tg positive. However, it has lower sensitivity and specificity for the diagnosis of 131I-Dx-WBS negative DTC and 18F-FDG PET/CT. The specificity increases with the increase of serum Tg level. The above results confirm that 18F-FDG PET/CT imaging is of great significance for the diagnosis of recurrence or metastasis in patients; with PET/CT imaging, the results changed 16.13% of the Tg-positive and 131I-Dx-WBS negative DTC patients' later treatment decision. The decision-making and curative effect evaluation have certain value.

## 1. Introduction

The superficial location of the thyroid gland makes it easy to find neck masses, and clinical palpation combined with neck B-ultrasound and puncture tissue biopsy are also easy to make a clear diagnosis [1]. There are many simple and easy methods for the differential diagnosis of benign and malignant goiters, and accurate staging of patients with thyroid cancer is a relatively difficult clinical problem. Modern surgery and head and neck tumor surgery are relatively mature. It is difficult to further improve the treatment effect of patients with thyroid cancer by improving surgical skills. Therefore, the location of preoperative metastases can further improve the efficacy [2]. Another problem that currently exists in clinical practice is the lack of specificity of neck dissection. Because the scope of neck dissection is too large, it increases the probability of postoperative dysfunction. Therefore, preoperative staging is helpful for targeted neck dissection, thereby reducing the incidence of postoperative complications which improves the quality of life of patients [3]. PET/CT is a new type of imaging equipment that has developed rapidly in recent years, and its value in the clinical staging of malignant tumors such as lung cancer, breast cancer, colon cancer, lymphoma, and malignant melanoma has been widely recognized [4]. The Health Care Financing Administration included FTC's PET staging in the scope of medical insurance payment, but other thyroid malignancies such as papillary cancer, medullary cancer, and undifferentiated thyroid cancer were not included. The diagnostic value of these thyroid cancers is still under discussion [5]. The diagnosis of thyroid cancer does not necessarily rely on PET/CT, but PET/CT itself requires the accumulation of experience in the diagnosis and differential diagnosis of thyroid cancer. For example, when PET/CT is used for health examination, it can be seen that the thyroid of some subjects is FIX [6].

Recent related work is described below. In recent years, 18F-FDG PET/CT whole-body imaging has been used to distinguish benign and malignant tumors, to detect curative effects, to detect metastases, and to determine prognosis, which has achieved important clinical value [7]. Thyroid hypermetabolic nodules, or incidental tumors, indicate high glucose metabolism and the presence of thyroid tumors, and it is also another important imaging method to show thyroid nodules [8]. According to reports in the literature, Beyer et al. [9] performed PET examinations on 4803 healthy physical examination populations and detected 60 cases of incidental thyroid tumors, with a detection rate of 1.2%. Yang et al. [10] counted 4,525 cases examined in the PET centers of three hospitals, and 71 cases of incidental thyroid tumors were found, with a detection rate of 1.6%. Huang et al. [11] reported that 999 cases of known tumor patients and 331 healthy volunteers underwent 18F-FDG PET/CT whole-body imaging and found that there were 19 cases and 10 cases of incidental thyroid tumors, and the detection rates were 1.9% and 3.0%, respectively. Shakeel et al. [12] retrospectively analyzed the 18F-FDG PET/CT whole-body imaging of 4136 subjects without a history of thyroid disease and found 45 cases (35 cases of women, 10 cases of men) of incidental thyroid tumors; the detection rate was 1.1%. The detection rate is higher than that of men (0.8%, 0.2%). Schöder [13] counted 1763 subjects who underwent 18F-FDG PET/CT examinations, found 70 cases of incidental thyroid tumors (the detection rate was 4.0%), and analyzed PET/CT examinations. However, in PET/CT, CT has a better positioning function and can provide more information. Liu et al. [14] performed 18F-FDG PET examination on 4,525 subjects, and 14 of 71 incidental tumors were pathologically diagnosed, of which 7 were malignant lesions, accounting for 50% of accidental tumors, 6 were high-functioning adenomas, and 1 was atypical hyperplasia of unknown origin. Lee and Lee [15] examined 1330 subjects with 18F-FDG PET and found 29 cases of incidental tumors, of which 15 cases were pathologically confirmed and 4 cases were malignant lesions, accounting for 26.7% of incidental tumors. Jager et al. [16] treated 4136 cases of thyroid incidental tumors in 45 cases without a history of thyroid disease. Among the 32 cases of pathological results, 16 cases were malignant lesions, accounting for 50% of incidental tumors. The reason for the relatively high thyroid cancer may be related to the examined population. Among the 16 malignant lesions, 14 cases were papillary carcinoma, and 2 cases were metastatic carcinomas of the breast and esophagus of origin; the other 16 cases were benign lesions, 2 cases were follicular tumors, 7 cases were nodular hyperplasia, and 7 cases were follicles of unknown nature [17–20]. Some scholars have reported that in the diagnosis of cervical UPT the probability of PET/CT detecting the primary lesion is 57%, PET + CT is 52%, and CT is only 23%, suggesting that PET/CT and PET + CT are in the diagnosis of UPT [21]. Some scholars reported that PET is better than CT and MRI in diagnosing UPT of primary lesions in the head and neck, but there is no significant difference between the two in chest tumors. FDG concentration may be false positive due to chest inflammation and tuberculosis [22]. Some researchers believe that PET does not have any advantages over CT and MRI. PET has its limitations in local tissue resolution and anatomical positioning compared to CT [23]. The application of PET/CT examination that combines anatomical and functional imaging examinations significantly reduces the false-negative and false-positive rates [24]. Some scholars found 70 cases of thyroid incidental tumors in 1763 18F-FDG PET and CT subjects. Among them, 49 patients obtained pathological results. 18 cases were found to be malignant tumors, accounting for 36.7% of incidental tumors, including 16 cases of papillary cancer. One case originated from esophageal cancer metastasis, and one case was NHL [25–27]. There have been several reports in the literature for many years [28–30]. However, PET/CT has the value of finding the primary tumor in patients with unidentified lymph node metastasis.

This subject conducts a retrospective analysis of patients undergoing PET/CT examinations, including some patients who are already aware of thyroid disease and are receiving thyroid hormone therapy. The purpose is to study 18F-FDG PET/CT whole-body imaging with diffuse thyroid uptake. The increased detection rate and its clinical significance can be suggested and known by clinical treatment. Because PET imaging can directly detect tumor foci through abnormalities in local metabolic activity, it has a higher specificity, which is helpful for the identification of other benign lesions, and can detect metastases in other organs and soft tissues at the same time, which is helpful to guide the clinical selection of a more appropriate treatment plan. The decision-making of treatment plan and the evaluation of curative effect have certain value. The sample size of this study is small and has certain limitations. Moreover, this study is a retrospective analysis. The factors that affect image quality in imaging methods are not standardized. This article retrospectively analyzes 18 groups in patients suspected of having bone metastases in routine imaging examinations. We analyze the PET/CT characteristics of different types of metastases and evaluate SUV in different types. For incidental cancers, both differentiated and undifferentiated thyroid cancers have high glucose metabolism changes; there is no statistically significant difference in the level of glucose metabolism in cancer foci of thyroid cancers with different levels of differentiation and invasion and metastasis.

## 2. Construction of a Precise Radiotherapy Model for Thyroid Cancer Based on PET-CT Fusion Deep Learning Imaging

### 2.1. PET-CT Imaging Level

PET is an imaging device that uses a tracer capable of emitting positrons to perform functional and metabolic imaging. It is characterized by high sensitivity and functional metabolic imaging. PET/CT is a composite function imaging device that combines PET and traditional imaging equipment CT. It can simultaneously obtain PET images which reflect the function and metabolic level of the lesion and CT images which reflect the anatomical structure in one examination.  Figure 1 shows the distribution of PET-CT imaging levels.

Diagnosis based on the metabolic difference between the diseased tissue and the normal tissue can detect and reflect the physiological, biochemical changes and metabolic abnormalities of the disease early, and the conventional method of PET imaging is whole-body tomography, which can show the distribution of the lesions on the overall level. In terms of scope, the PET/CT fusion image can obtain the abundant functional information of the molecular metabolism of the lesion, and at the same time, it can accurately locate the lesion and clarify the violation of the surrounding soft tissues, realizing the simultaneous fusion of molecular and anatomical images:

(1) $$\begin{array}{c} a\left[n\right]=\left\{a1,a2,\ldots ,an\right\},\;\left(n=1,2,\ldots ,i\right). \end{array}$$

Therefore, the use of PET/CT imaging by FDG can reflect the uptake and utilization of glucose by the lesions in the body and provide image information of the glucose metabolism capacity of the lesions. FDG in the blood is transported into the cell by GLUTs (mainly GLUT-1) located on the cell membrane and then formed under the catalysis of hexokinase (HK), which cannot be further metabolized by enzymes in the cell.

(2) $$\begin{array}{c} u\left(i,j\right)=s^{T}\tanh\left(s\left(i\right)\times a\left[i\right]\right). \end{array}$$

The amount of 6-P “accumulated” in the cell is consistent with the ability of the diseased cells to take up and use glucose. The amount of P can reflect the demand for glucose by the lesion, because most malignant tumors in the body have abnormally upregulated uptake and utilization of glucose. After lying supine in the dark room for 50–60 minutes, PET/CT imaging of the body was performed, and each bed was collected for 3 minutes with a thickness of 5 mm. Image reconstruction adopts the maximum expected value iteration method of ordered subsets to obtain three-dimensional images and cross-sectional, coronal, and sagittal tomographic images:

(3) $$\begin{array}{c} \frac{v\left(x\right)}{\alpha \left(i\right)}=\text{soft}\max\left(u\left(i,j\right)\times k\left(x\right)\right). \end{array}$$

Therefore, whether there is abnormally increased FDG concentration in the lesion on the PET/CT image can reflect whether the sugar metabolism of the diseased cell is abnormally increased, and PET/CT imaging can diagnose the benign and malignant nature of the lesion. SUV is a semiquantitative index that reflects the concentration of imaging drugs in the lesion on PET imaging. It is generally believed that SUV is more likely to be malignant lesions above 2.5–3.0, and benign lesions below 2.0 are likely larger, and between these two values, the benign and malignant quality of the lesion cannot be determined, and it is classified as a suspicious lesion:

(4) $$\begin{array}{c} \frac{\langle m\left|x\right|n\rangle }{\langle m|n\rangle }=\int \int u\left(x\right)\times v\left(x\right)\times du\times dv. \end{array}$$

Through visual analysis, the distribution of 18F-FDG in the thyroid region is higher than that of the surrounding normal thyroid tissue, which is a focal hypertrophy of thyroid. For selecting the most significant level of uptake by thyroid lesions, the region of interest (ROI, 1.0 cm in diameter) technique was used to determine the maximum standard uptake value (SUVmax) of lesions and regional lymph node measurement lesions. SUV value is an important parameter for 18F-FDG PET/CT imaging to evaluate the glucose metabolism of lesions. The SUV value of malignant tumor tissue will increase, and the SUV value of normal thyroid tissue will not increase. Semantic segmentation information is fused to points through the transformation matrix of lidar information and image information, and then baseline object detection is used; it can be understood that the semantically segmented objects have more information as a guide to obtain better detection accuracy. The fusion is a tandem network structure that sends the semantically segmented features and the original point cloud into the deep learning network. In this study, the SUV value of incidental thyroid cancer foci was significantly higher than that of normal thyroid tissue:

(5) $$\begin{array}{c} \left[\begin{array}{cc} x1 & 0\\ 0 & xn \end{array}\right]=\left[\begin{array}{cc} \cos\left(x\right) & \sin\left(x\right) \end{array}\right]\times \left[\begin{array}{c} f\left(x\right)\\ f^{-1}\left(x\right) \end{array}\right]. \end{array}$$

The determination of the concentration of the lesion tracer on the PET image adopts a combination of visual analysis and semiquantitative analysis, namely, standard uptake value (SUV) measurement, combined with the corresponding level of low-dose CT image and the fusion of the two images to judge the benign and malignant lesions. (1) CT image features include lesion location, size, density, edge, shape, and relationship with adjacent tissues; (2) PET image features, in addition to SUV value, refer to the size, shape, and edge of the tracer distribution area and the uniformity of the tracer distribution, etc. The results of PET/CT were visually analyzed and semiquantitatively analyzed.

(6) $$\begin{array}{c} g\left(x\right)=\frac{1}{\sqrt{N}}\times \sum \sum \exp\left(ikx\right)\times f\left(x\right), \end{array}$$

(7) $$\begin{array}{c} \frac{\partial y\left(x\right)}{\partial x}+\frac{\partial y\left(x\right)}{\partial y}+\frac{\partial y\left(x\right)}{\partial z}=e. \end{array}$$

SPSS 19.0 statistical software was used to analyze the data. The measurement data is expressed by *x* ± *s*, the mean comparison is performed by *t*-test, the correlation analysis is performed by Person correlation analysis, and the comparison of rates is performed by the *χ*2 test. *P* < 0.05 indicates that the difference is statistically significant. At the same time, the SUVmax of normal thyroid tissue was measured. The diameter of the thyroid lesion was measured by CT image.

(8) $$\begin{array}{c} \left\{\begin{array}{cc} h\wedge \frac{2}{\left(2*m\right)}-z\left(k-k0\right)=0, & k>k0,\\ \int \frac{z\left(k\right)}{m}*\text{d}s=0, & k<k0. \end{array}\right. \end{array}$$

In this study, the SUVmax values of differentiated thyroid cancer, medullary cancer, and poorly differentiated cancer were 4.25 ± 1.70 and 6.34 ± 2.45, respectively. The SUV values of medullary cancer and poorly differentiated cancer were slightly higher than those of differentiated thyroid cancer, but there was no difference.

### 2.2. Deep Learning Fusion Algorithm

Eligibility criteria for increased thyroid 18F-FDG uptake are as follows: confirmed by two experienced nuclear medicine doctors, the patient can see the two lobes of the thyroid in the three-dimensional MIP image. Theoretically speaking, the image information is dense and regular, including richness. Relative to the image, the expression of the point cloud is sparse and irregular, which makes it infeasible to directly process the point cloud using traditional perception. But the point cloud contains three-dimensional geometric structure and depth information, which is more beneficial for 3D target detection, so the two kinds of information are theoretically complementary. In addition, in the current two-dimensional image detection, deep learning methods are all based on it. Manually, we measure the degree of concentration, adjust the background to the liver brightness level, and measure the thyroid uptake on the cross-sectional PET/CT fusion image. Semiquantitative analysis of diffuse thyroid uptake: the same operator carefully delineates the region of interest (ROI) and places it at the highest point of thyroid uptake of 18F-FDG. The computer automatically calculates the intake SUVmax and selects the two leaves. On the cross-sectional image, we select the level with the highest radioactive concentration of the lesion with abnormal visual analysis and use the region of interest (ROI) method to measure the maximum standardized uptake value of the lesion. The ROI includes 2/3 of the tumor cross-sectional area.  Figure 2 shows the flow of the deep learning fusion algorithm. If there is no abnormal concentration of radioactivity on PET imaging, according to the same CT or the patient's conventional CT, MRI, the location of the lesion is shown, and the method of visual fusion is used to delineate the ROI of the same size as the lesion in the corresponding part.

The image analysis is performed by two experienced nuclear medicine doctors who jointly and independently read the diagnosis. When the conclusions are inconsistent, the results after discussion are used as the final diagnosis. DTC patients undergoing 131I-WBS after thyroid surgery and 131 treatment usually have normal radioactive accumulation sites: salivary glands, nasopharynx, gastrointestinal tract, and bladder. 131I-WBS image analysis excludes physiological uptake and radioactive contamination of normal tissues and locates and qualitatively diagnoses lesions with abnormal radioactive uptake. The acquisition range is from the base of the skull to the middle part of the femur. Spiral CT scan and then PET image acquisition are performed in 3D mode. The acquisition time for each bed is 5 minutes. Attenuation correction is performed on the image, and the axial, coronal, sagittal, and MIP images are obtained after iterative reconstruction, and the CT and PET images are fused. Image analysis is performed by two experienced PET/CT physicians who independently read the film for diagnosis and reached a consensus as the final diagnosis.

### 2.3. Optimization of Radiotherapy Model Indicators

PET/CT imaging of 18F-FDG, 18F-FCH, and 18F-FMISO are three imaging agents: ① take 18F-FDG and 18F at the transplanted tumor site on PET/CT imaging FCH, in which 18F-FDG uptake is larger than 18F-FCH; 18F-FMISO has no obvious uptake; all three imaging agents in inflamed tissues are ingested. The SUVmean of 18F-FDG, 18F-FCH, and 18F-FMISO uptake by xenograft tumors was about 7.58 ± 1.05, 3.19 ± 0.38, and 1.05 ± 0.41, respectively, and the difference was statistically significant by paired *t*-test (18F-FDG group and 18F-FCH group).

② In addition to tumor and inflammatory tissue uptake, 18F-FDG PET/CT showed that the uptake of 18F-FDG in the brain, kidney, and liver of nude mice was significantly increased; 18F-FCH PET/CT showed that 18F-FCH was in the kidney and the liver of nude mice. The uptake of the liver was significantly increased; 18F-FMISO PET/CT showed that the uptake of 18F-FMISO in the liver and kidney was significantly increased.  Figure 3 shows the histogram of standard uptake values for different cases. ③ The three groups of imaging agent tumor and muscle SUVmean ratio (T/NT) from high to low are FDG group > FCH group > FMISO group, FDG group and FCH group, FDG group and FMISO group, FCH group and FIMSO group *t*. The values are 6.214, 10.159, and 6.842; *P* values are 0.05; the three groups of imaging agent tumor and lung SUVmean ratio (T/NT) from high to low are FDG group > FCH group > FMISO, FDG group and FCH group, FDG group and FMISO group, FCH group, and FIMSO group *t* values were 7.245, 10.365, and 5.968, respectively; *P* values were 0.05; the SUVmean ratios (T/NT) of the three groups of imaging agent tumor and inflammatory tissues from high to low are FCH group > FDG group > FMISO group, FCH group and FDG group, FDG group and FMISO group, FCH group, and FIMSO group *t*. The values were 7.124, 9.982, and 6358, respectively, and the *P* values were 0.001.

## 3. Application and Analysis of the Precise Radiotherapy Model for Thyroid Cancer Based on PET-CT Fusion Deep Learning Imaging

### 3.1. PET-CT Data Preprocessing

The instrument used is Aplio XG color Doppler ultrasound produced by TOSHIBA company or 22 color Doppler ultrasound produced by Philips company. The patient was in a supine position, and the neck was fully exposed at the same time, and the thyroid and bilateral cervical lymph nodes were explored in a certain sequence. In this article, 27 cases of thyroid 18F-FDG uptake increased SUV max ranging from 2.40 to 7.80, mean 4.1 ± 1.3. After culturing for another 15 days in the irradiation group for 24 h, the clone formation rate was (90.13 ± 7.76)%, while that of the control group was (74.60 ± 6.96)%. Western Blot was used to determine the expression of three thyroid-specific proteins TSHR, NIS, and TPO in K1 cells after 24 hours of low-dose 131I radiation and in K1 cells without radiation.  Figure 4 shows the precise radiotherapy model framework for thyroid cancer based on PET-CT fusion deep learning imaging.

Seventy-nine patients who did not take 18F-FDG were randomly selected for thyroid PET/CT examination. There were 49 females and 30 males. Gender, age, and clinical conditions matched those of the study group, and there was no statistically significant difference. Clinical data: 30 cases of tumor or tumor screening, 2 cases of tumor marker CA199 elevated, 2 cases of Graves' patients, 3 cases of hypothyroidism patients, and the rest were patients on physical examination. From 79 cases of PET/CT examination of thyroid with no 18F-FDG uptake, 56 cases of US and thyroid laboratory examination were selected. The findings of thyroid US examination are as follows: 10 cases of diffuse thyroid disease, 15 cases of thyroid nodular disease, 8 cases of diffuse thyroid nodular disease, 3 cases of unilateral thyroid nodule, and 20 cases of bilateral thyroid no abnormalities.  Figure 5 shows the comparison curve of the test and control lesion rates of different sample groups. The statistical results showed that the difference between the experimental group and the control group was statistically significant (*t* = 17.84, *P* = 0.00), suggesting the difference in the metabolic mechanism of the disease and confirming the SUV through the disease. The test method is feasible. Both groups of K1 cells had the expression of TSHR protein, NIS protein, and TPO protein, but compared with the control group, the expression level of the 24 h radiation group was significantly reduced.

After the image was processed by the analysis software, the expression levels of TSHR, NIS, and TPO relative to *β*-actin in the 24-hour radiation group were 0.34 ± 0.025, 0.25 ± 0.02, and 0.37 ± 0.01, respectively, while the TSHR, NIS, and TPO of K1 cells in the control group were relatively larger. The expression levels of *β*-actin were 0.52 ± 0.02, 0.45 ± 0.03, and 0.63 ± 0.02. The comparison between the two groups was *P* < 0.001. After 24 hours of low-dose 131I irradiation, the expression of the three proteins characteristic of differentiated thyroid cancer decreased, suggesting that after 24 hours of low-dose 131I irradiation, K1 cells transformed into low/dedifferentiated thyroid cancer cells.

### 3.2. Realization of Deep Learning Visualization Simulation

In this study, if SUV = 2.5 is used as the cut-off value for the diagnosis of benign and malignant thyroid, the sensitivity for the diagnosis of primary tumor is 96.67%, and the specificity is only 45.45%; if SUV = 3.0 is the diagnostic critical value, the sensitivity is 86.67%, and the specificity is 72.73%. The latter is more suitable as the cut-off value for the diagnosis of benign and malignant lesions. If time-lapse imaging technology can be supplemented at the same time, it will definitely help to further improve the specificity. This study found that if SUV = 2.5, as the cut-off value for benign and malignant diagnosis, PET/CT used in the differential diagnosis of thyroid cancer has the characteristics of high sensitivity and low specificity.  Figure 6 shows the dependence of imaging sensitivity under deep learning on the level of radiotherapy. PET/CT detected a total of 483 osteolytic metastases, SUV was 9.21 + 4.46, 374 osteogenic metastases, and SUV product was 3.80–1.56. The SUV difference between osteolytic metastasis and osteogenic metastasis was statistically significant (*t* = 19.49, *P* < 0.001).

Due to limited conditions, the number of samples of benign lesions in this study is small and the types of lesions are small, and it fails to include benign thyroid adenoma and other benign thyroid lesions. When PET/CT diagnoses thyroid cancer, some benign thyroid lesions will affect its diagnostic accuracy. In 16 patients, 996 abnormal lesions were detected by PET/CT. The SUV ranged from 1.3 to 14.0, with an average of 4.1 ± 1.9. Excluding MM, the other 9 cases of bone primary malignant tumors detected 11 lesions. The SUV ranged from 2.7 to 27.1, with an average value of 13.1 + 8.0. The difference in SUV between the two groups was statistically significant (net = 3 .73, *P* = 0.04). The FDG group was significantly higher than the FCH group and the FMISO group, but the FCH group and the FMISO group were only slightly increased.  Figure 7 shows the response curve of the specific deviation level over time. The SUVmean ratio (T/NT) of the three groups of imaging agents from high to low was FCH group > FDG group > FMISO group. The above studies have shown that PET can detect the treatment response group and the ineffective group more sensitively than CT. The reason may be that metabolic changes after tumor treatment are more sensitive than morphological changes, and PET can precisely detect this kind of change. The FCH group was significantly higher than the FDG and FMISO groups, while the FDG group was only slightly higher.

The Smirnov test showed a normal distribution (*P* = 0.520), and the reciprocal of the time-lapse imaging SUV also showed a normal distribution (*P* = 0.487, *P* = 0.605). The paired *t*-test was used to test the significant differences between the means of lesion 1/SUV and delayed 1/SUV in groups, respectively.  Figure 8 shows the two-dimensional scatter distribution of imaging correlation coefficients for different radiation dose ratios. The results suggest that the time-lapse imaging SUV in group was significantly higher than the conventional imaging SUV, while there was no significant difference between groups time-lapse imaging SUV and conventional imaging SUV (*t* = 1.855, *P* = 0.123).

Time-lapse imaging was performed on 16 thyroid cancer lesions in group, 87.5% (14/16) of the lesions with delayed imaging SUV were higher than conventional imaging SUV, and the increase range was 7.89%～37.32%. In this study, 16 cases of myeloma lesions were compared with 11 cases of bone primary malignant tumors in SUV and it was found that the difference between the two was statistically significant (*t* = 3.73, *P* = 0.04). This shows the difference in FDG metabolism between bone marrow tumors and other bone malignancies. On the other hand, 12.5% (2/16) of the lesions experienced a decrease in the SUV of delayed imaging, and the decrease range was from 2.94% to 10.66%. Time-lapse imaging was performed on 6 benign lesions in group, of which 83.33% (5/61) time-lapse imaging SUV showed a decrease; the decrease range was 7.41%–44.74%, and 16.67%. Time-lapse imaging SUV showed an increase; the increase rate was 10.53%.

### 3.3. Example Application and Analysis

The SUV of the thyroid cancer group was significantly higher than that of the benign lesion group, and the two groups of benign and malignant lesions were higher than the normal control group. There is no significant correlation between the SUV of the primary thyroid cancer and the SUV of the metastasis, while the volume of the primary thyroid cancer has a significant positive correlation with the SUV of the lesion. Delayed imaging of thyroid cancer SUV is significantly higher than conventional imaging, but benign lesions do not have this feature, so it is believed that this feature is helpful for the differentiation of benign and malignant thyroid lesions. If SUV = 2.5 is used as the critical value for the diagnosis of thyroid benign and malignant lesions, it has the characteristics of high sensitivity and low specificity, and it needs to be combined with time-lapse imaging technology to enhance specificity. Taking SUV = 3.0 as the cut-off value is more suitable for the diagnosis of thyroid cancer. The specificity of the diagnosis is improved but the sensitivity is reduced. Comparison of SUV between malignant bone lesions and benign lesions: in 101 patients in this study, a total of 1864 bone malignant lesions were detected by PET/CT, SUV forging was 5.54–3.8, benign lesions were 96, and SUVm was 5.7–3.6; statistical analysis showed that the difference between the two groups was not statistically significant (*t* = 0.39, *P* = 0.70).  Figure 9 shows the error statistics box plots for different sample groups. Among 1,864 bone malignant lesions detected by PET/CT, 857 bone metastases had SUV = 7.2–4.5. There were 1007 primary malignant tumor lesions, and the SUV ranged from 4.24 to 2.4.

There are reports in the literature that increased 18F-FDG uptake in thyroiditis is related to lymphocyte infiltration. For example, it is reported that, among 4,732 cases, 2.9% of 138 cases showed diffuse thyroid uptake, and 63 cases (47.4%) of 133 cases were diagnosed with hypothyroidism. In this article, except for the diagnosis of hypothyroidism or chronic thyroiditis, although there is no pathological diagnosis in other cases, there are more people with positive antithyroid antibodies, so it may be related to thyroiditis.  Figure 10 shows the PET-CT imaging sensitivity matchstick chart for different data points. In this study, the three imaging agents uptake 18F-FDG and 18F-FCH at the transplanted tumor site on PET/CT imaging.

The tumor and muscle SUVmean ratios (T/NT) of the three groups of imaging agents from high to low are FCH group > FDG group > FMISO group, of which the FCH group is slightly higher than the FDG group, and both the FCH group and the FDG group are significantly higher than FMISO. FCH group is significantly higher than FDG group and FMISO group while FDG group is only slightly higher than the FMISO group. It explained that 18F-FDG PET/CT imaging has high resolution and image quality.  Figure 11 shows the data fitting curve of the disease detection rate. The results show that it has high sensitivity but low specificity and false positives. The specificity and sensitivity of 18F-FCH imaging indicate that it is an ideal imaging agent, while 18F-FMISO is not an ideal imaging agent.

According to Kolmogorov–Smirnov test, the thyroid SUVs of the three groups showed a normal distribution, but the variance among the three groups was not uniform; after the reciprocal transformation of the SUV of each group, the variance was uniform (Levene Statistic is 0.42), and after statistical processing, the three groups were asked about the thyroid SUV. Grouped by pathological type, the SUV of the lesions is normally distributed, but the homogeneity of variance test shows that the variance is uneven; the variance is equal after the reciprocal conversion (statistic is 0.769, *P* = 0.575). Since there is only 1 case of squamous cell carcinoma in the tumor group, it cannot be included in the statistics and therefore did not participate in further analysis. 1/SUV is a variable for analysis of variance, which indicates that there are significant differences between the groups, indicating that there are significant differences between the groups.  Figure 12 shows the histogram of the confidence interval of the lesions at different sample points. The mean of each group is compared in pairs. There are significant differences between the means of any two groups of three groups (*P* = 0.001), and the SUVs of the control group, benign lesion group, and thyroid cancer group increased in turn.

Comparison of SUV among three groups of different types of bone lesions: 50 cases of bone metastases with PET/CT detected a total of 857 lesions, 374 osteogenic metastases, SUV of 3.8 ± 1.6. There were 438 foci, and the SUV was 9.21 ± 4.5. A total of 1,007 foci were detected in 25 patients with primary bone malignancies, including 996 multiple myeloma and SUV. The cough was 4.1 ± 1.9, the remaining bone primary malignant tumors were 11 lesions, and the SUV was 13.1 ± 8.0. A total of 96 lesions and 34 lesions were detected in 26 patients with benign lesions. Although the standard results are consistent, the PET-based metabolic evaluation criteria are more accurate in predicting the effect of treatment and may be more suitable for the evaluation of the efficacy of targeted therapies than the morphological evaluation criteria.

## 4. Conclusion

In this paper, 18F-FDG and 18F-FCH were taken in the tumor site on PET/CT imaging, and 18F-FMISO was not significantly taken up; all three imaging agents were taken in inflammatory tissue. 18F-FDG has high sensitivity in diagnosing recurrence or metastasis, but its specificity is poor. 18F-FCH may be a useful supplement to 18F-FDG PET/CT imaging, and case studies need to be further expanded. However, the results of this study show that the SUVmax of the primary thyroid cancer is not statistically different between the metastatic group and the nonmetastatic group. The evaluation metabolic parameters we use are different from them, which may lead to differences in the results of the study. Therefore, it is necessary to expand the sample size and use a variety of parameters for evaluating glucose metabolism to conduct research in this area. This study shows that the SUVmax of thyroid cancer is positively correlated with the size of the lesion. Studies have reported that the size of the lesion is one of the important factors affecting the SUV value. In this study, 8 cases of thyroid microcarcinoma were not developed on 18F-FDG PET/CT imaging because the small lesions were affected by the imaging resolution limitation or partial volume effect. It can be seen that 18F-FDG PET/CT imaging is of great significance for the detection of recurrence or metastasis in patients with Tg-positive and 131I-Dx-WBS-negative DTC.

## Figures and Tables

**Figure 1:** The layered distribution of PET-CT imaging.

**Figure 2:** Deep learning fusion algorithm flow.

**Figure 3:** Histogram of standard uptake values for different cases.

**Figure 4:** The framework of a precise radiotherapy model for thyroid cancer based on PET-CT fusion deep learning imaging.

**Figure 5:** Comparison curves of test and control lesion rates of different sample groups.

**Figure 6:** The dependence of imaging sensitivity under deep learning on the level of radiotherapy.

**Figure 7:** Response curve of a specific deviation level over time.

**Figure 8:** Two-dimensional scatter distribution of imaging correlation coefficients for different radiation dose ratios.

**Figure 9:** Box plot of error statistics for different sample groups.

**Figure 10:** PET-CT imaging sensitivity matchstick chart for different data points.

**Figure 11:** Data fitting curve of the disease detection rate.

**Figure 12:** The histogram of the confidence interval of the lesion for different sample points.

## Data Availability

Relevant data are available from the corresponding author upon request.
